# Investigation on the Correlation of Anxiety Degree with Family Atmosphere in Children with Precocious Puberty

This article has been retracted.

**DOI:** 10.1155/2022/3269807

**Published:** 2022-09-23

**Authors:** Yongbei Xiao, Yamin Li, Zhengrong Cai, Jiao Xie

**Affiliations:** ^1^Clinical Nursing Teaching and Research Section, The Second Xiangya Hospital, Central South University, Changsha 410011, Hunan, China; ^2^Department of Pediatrics, The Second Xiangya Hospital, Central South University, Changsha 410011, Hunan, China

## Abstract

**Objective:**

This research sets out to explore the correlation of anxiety degree with family atmosphere in children with precocious puberty (PP), so as to provide a reference for future treatment of PP.

**Methods:**

Eighty-one cases of PP were visited between January 2021 and March 2021, and their direct relatives were selected as the research population for retrospective analysis. After admission, children and their direct relatives completed a questionnaire survey on the quality of life and social anxiety of children with PP. Children were assigned to the research group and the control group based on their anxiety scores. The intergroup differences in daily activities, diet, and family status, as well as children's and parents' psychological status, were identified, and the relationship between anxiety degree in PP children and family atmosphere was discussed.

**Results:**

The children's anxiety score was (6.17 ± 4.26), and they were divided into groups according to the median, with 30 cases in the research group and 51 cases in the control group. The two cohorts were similar in dietary status and children's physiological status (*P* > 0.05); however, the research group exhibited a greater number of cases who used electronic products for 2-3 h daily and watched romantic TV series (movies). The daily exercise time of the research group is lower than that of the control group (*P* < 0.05). In the research group, the monthly family income and the number of family companions and very harmonious families were significantly lower, while the number of divorces or remarriages increased (*P* < 0.05). The survey results on parents' psychological status also showed better psychological states in patients in the control group (*P* < 0.05).

**Conclusion:**

The anxiety level of PP children is closely related to the family atmosphere. In future clinical treatment of children with PP, it will also be necessary to pay attention to and adjust the family relationship of the children, which is of great significance for relieving PP-associated anxiety.

## 1. Introduction

Precocious puberty (PP) is an endocrine disease with abnormal growth and development in children, which refers to the presentation of secondary sexual characteristics in girls before the age of 8 and boys before the age of 9, more common in girls [1]. For example, the symptoms of girls are more rapid breast development than their peers and the appearance of axillary hair, pubic hair, and menophania, while the symptoms of boys mostly include increased testicular volume, an enlarged penis, a beard, pubic hair, and so on [2]. Current clinical data show an increasingly high incidence of PP due to various reasons, such as the popularization of modern Internet information [3]. In some developed countries, PP is more common, and the incidence of urban children is significantly higher than that of rural children [4]. In addition to the seriously affected physical development of children due to the occurrence of PP, the long treatment process may greatly cause adverse effects on children's psychology, leading to anxiety and depression; while parents, as relatives, are also susceptible to anxiety and psychological pressure when facing the treatment of their children, which eventually leads to family disharmony [5].

In the prevention and treatment of modern PP, it is usually necessary to provide psychological counseling to children so that they can view PP correctly [6]. Common methods include explaining the knowledge of precocious puberty to children, encouraging children to maintain an optimistic and cheerful attitude, etc. [7, 8]. It is not difficult to find that the current psychological counseling on PP is more concerned with children, and with the limited information available regarding the issue, it ignores the relationship between children and their family atmosphere. We believe that understanding the relationship between the psychological state and family atmosphere of PP children is the basis of psychological relief therapy. Psychological research points out that improving the quality of life of children and their families and the degree of family harmony can effectively promote children's physical and mental health during their growth [9, 10]. It can be seen that when providing psychological counseling for children with PP, it is also necessary to pay attention to the influence of the family atmosphere. Since 2021, our hospital has launched a survey and research on the family atmosphere of children with PP admitted to our hospital, and a sufficient number of cases have been accumulated so far. Therefore, in this study, we will summarize and report the characteristics of such PP children, and analyze the relationship between the anxiety level of children and family atmosphere, aiming to provide reliable evidence for future clinical prevention and treatment of PP children.

## 2. Materials and Methods

### 2.1. Research Participants

A retrospective analysis was performed on 81 PP children admitted between January 2021 and March 2021 and their immediate family members. Based on the median anxiety score, children with a score ≥ median were assigned to the research group, and those with a score < median were set as the control group. Patients' basic information, such as age and sex, is shown in Table 1. This study was carried out in strict accordance with the guidelines laid down in the Declaration of Helsinki, and all the legal guardians of the research subjects signed the informed consent.

### 2.2. Eligibility Criteria

Children enrolled in the research group all conformed to the diagnostic guidelines for PP [11] and were diagnosed as PP by clinical trials in our hospital, requiring long-term gonadotropin-releasing hormone therapy; moreover, the children and their immediate family members had good communication skills and could cooperate to complete the investigation. Children with organ disorders such as liver, lung, and brain, unfixed primary caregivers, other endocrine diseases, congenital defects or disorders, and mental diseases were excluded. children who underwent physical examination in our hospital, with normal physical examination results, no major physical or psychological history and good communication skills, and willingness to cooperate with the investigation were included in the control group.

### 2.3. Evaluation Tool

After admission, the research subjects, accompanied by their parents, completed a questionnaire survey on the quality of life and social anxiety in children with PP (https://www.wjx.cn/xz/105367013.aspx). The survey was divided into six items, including five items answered by parents (including basic information, daily activities, diet, family status, and physiological status of children) and one item answered by children (an anxiety level survey). The children answered a total of 10 questions, and the alternative results were never (0), sometimes (1 point), and always (2 points), for a full score of 20. The higher the score, the more serious the child's anxiety.

### 2.4. Investigation Methods

After the subjects were admitted to the hospital, a questionnaire survey was conducted through WeChat. Before they filled it out, the investigator carefully explained the purpose and content of the survey to the subjects. If the subjects had a reading or filling-in obstacle, the investigator would dictate the relevant contents for them and then let the subjects make their own choices. After completing the survey, the scale was submitted on the spot and filed by the researcher on the computer. The children's answers were sorted out separately, and the final anxiety score was counted.

### 2.5. Statistics and Methods

Data processing was carried out by SPSS24.0. A chi-square test was performed for the intergroup comparison of the categorical data recorded in the form of [*n* (%)]. The quantitative data were expressed as ($\bar{\chi }\pm s$). Statistical significance was present when *P* < 0.05.

## 3. Results

### 3.1. Grouping

In this experiment, all the children's anxiety scores were (6.17 ± 4.26), and they were grouped according to the median, including 30 cases in the research group and 51 (score ≥6) cases in the control group (score <6). Comparing the anxiety scores of the two groups, it can be seen that the anxiety score of the research group was (8.53 ± 2.08), which was significantly higher than that of the control group (2.37 ± 1.77), *P* < 0.001.  Figure 1

### 3.2. Comparison of Children's Daily Activities

First of all, we compared the survey results related to children's daily activities. The results showed no intergroup differences in total sleeping time, sleep with lights on at night, time spent outdoors, sports items, and the use of adult skin care products (or cosmetics) between the control group and the research group (*P* > 0.05). However, the use time of the research group on electronic products and the number of people who have watched romantic TV series (movies) are significantly more than the control group, and their daily exercise time is less than the control group (*P* < 0.05).  Table 2

### 3.3. Comparison of Diet

Then, comparing the diet structure, it can be seen that the two cohorts of children also differed insignificantly in feeding patterns, eating habits, food intake, and frequency of drinking milk before half a year old (*P* > 0.05).  Table 3

### 3.4. Comparison of Family Status

The intergroup comparison of family status revealed no obvious difference in parents' education level and occupation as well as children's living environment (*P* > 0.05); however, the monthly income and family companionship of the research group were obviously less compared with the control group, with fewer numbers of very harmonious families and a higher number of divorces or remarriages (*P* < 0.05).  Table 4

### 3.5. Comparison of Children's Physiological Status

According to the intergroup comparison of children's physiological status, the research group was not statistically different from the control group in the survey results of running, participating in sports or exercise, lifting heavy objects, doing housework, injury, and poor physical strength (*P* > 0.05).  Table 5

### 3.6. Comparison of Parents' Psychological States

Comparing parents' psychological states, it can be seen that the parents' psychological states in the research group were significantly worse compared with the control group (*P* < 0.05), which shows that the parents of the research group had more obvious unhealthy psychological states and negative emotions.  Table 6

## 4. Discussion

PP is a very common childhood disease. Because of the influence of sex hormones, children's epiphyseal lines will close early, resulting in height retardation [12]. Besides, some PP girls may have early sexual behaviors due to the mismatch between psychological development and physical development, lack of life experience, and poor self-control, which may have a certain impact on their future fertility [13]. Moreover, children with PP generally have great psychological barriers, which directly affect their normal life, study, and family relations and may even lead to endocrine disorders [14]. Therefore, timely and effective improvement of PP is of great significance for the normal growth of children.

In this study, we made a preliminary analysis of a questionnaire survey targeting PP children and compared the differences between PP children and normal children from many aspects. First of all, in daily life comparison, the research group spent significantly less time exercising and significantly more time using electronic products and watching romantic TV series, which is consistent with our expectation that we believe is due to psychological disorders. As we all know, proper physical exercise can effectively accelerate the secretion of growth hormones in the process of children's development, which can enhance their self-confidence and hard-working spirit while improving body function [15]. A study shows that children with PP will resist sports because of their psychological inferiority and fear of socializing, and choose to be alone or indulge in online virtual worlds [16]. This also agrees with the findings of this survey, indicating that one of the basic conditions for improving PP is to increase physical exercise and improve children's communicative ability. Second, the intergroup comparison of eating habits showed no obvious differences, indicating a nonsignificant influence of diet on PP. However, Pollom TR et al. proposed that children's diets should be based on high protein and vitamins, with a reasonable combination of meat and vegetables, which will help children to grow and develop better [17]. Excessive intake of oils and fats, on the contrary, may lead to obesity and endocrine disorders in children, which may also affect the secretion of sex hormones to a certain extent [18]. Therefore, although this study indicates no significant effect of diets on PP, we still need to pay attention to the reasonable collocation of children's diets. Subsequently, in the comparison of children's family status, it can be seen that the family's monthly income and the number of family companionships and very harmonious families were statistically lower in the research group, while the number of divorces or remarriages were higher, which indicates that family status has a very close relationship with the anxiety level of PP children. We believe that in the follow-up treatment of PP children, it is also necessary to pay attention to the health education of the children's families. On the one hand, it is clinically necessary to guide children to face the disease with a positive attitude. Meanwhile, strengthening communication with the families of PP children, urging parents to pay more attention to the psychological changes of children, and strengthening communication among family members are essential. In addition, medical bulletin boards can be used to popularize relevant knowledge among the public, improve social support, and boost the quality of life of children and their families. Similarly, in previous studies, it was also mentioned that when the children's family atmosphere is poor and their illness cannot be supported by their families, the two parties cannot have a positive resonance, which will increase children's negative psychological emotions and parents' parenting pressure [19]. In contrast, in a harmonious family, children are more willing to share their ideas with their parents, and parents can understand and support each other well, which is beneficial for both sides to establish benign behaviors and improve the ability to solve family problems [20]. Furthermore, the two cohorts of children exhibited no obvious difference in physiological states, which shows that the main influence of PP-induced anxiety has nothing to do with the patients' physiological conditions, similar to the results of previous studies [21]. The reason for the lack of a significant difference between the two groups may be that the occurrence of PP does not affect the normal physiological function of children. Therefore, there is no difference in physical function among children with PP with different anxiety levels. It may also be because the children with PP included in this study did not have any malignant pathological diseases due to PP, so their physical activity remained in a normal state. In view of this situation, we will confirm the life activity level of children with intracranial mass effects caused by PP in the future. Finally, in the investigation of parents' psychological states, we found notably better psychological states in parents in the control group, which also verifies our view, that is, there are mutual influences between PP children and their families. A good family atmosphere can alleviate the anxiety of PP children and even effectively prevent PP. While a bad family atmosphere may further promote the progression of PP and can bring greater burden and pressure to families with the increased severity of PP, further worsening the family atmosphere and forming a vicious circle. Therefore, the key to alleviating the anxiety of PP children also lies in how to adjust the atmosphere for the children and their families. At the same time, it is also necessary to strengthen children's outdoor physical exercise, reduce the use time of electronic products, and establish a sunny, positive, and cheerful atmosphere for children's growth, thereby reducing the possibility of PP.

Of course, this research also has many limitations to be addressed. For example, this study is a retrospective analysis with many uncertain and uncontrollable factors, which may result in some contingency, requiring randomized controlled trials for validation as soon as possible. Second, we need to obtain more representative results by expanding the number of research participants. Third, the children enrolled need to be followed up for a longer time to further evaluate their long-term prognosis.

All in all, the anxiety level of PP children is closely related to the family atmosphere. In future clinical treatment of children with PP, it will also be necessary to pay attention to and adjust the family relationship of the children, which is of great significance for relieving PP-associated anxiety.

## Figures and Tables

**Figure 1:** Comparison of anxiety scores between study and control groups. ^*∗∗∗*^*P* < 0.001.

**Table 1:** Basic information of precocious puberty children.

Project	Data
Age	8.31 ± 1.58
Height (cm)	137.12 ± 8.95
Weight (kg)	32.45 ± 6.36
Gender	
Boy	4 (4.94)
Girl	77 (95.06)
Type of drug therapy	
Two or more	28 (34.57)
Not receiving treatment	21 (25.93)
Only one drug	30 (37.04)
Traditional Chinese and western medicine	2 (2.47)
Drug treatment route	
Subcutaneous injection	39 (48.15)
Intramuscular injection	8 (9.88)
Both	12 (14.81)
None	22 (27.16)
Living environment	
City	59 (72.84)
Rural or township	22 (27.16)

**Table 2:** Survey results of children's daily activities.

Project	Control group (*n* = 51)	Research group (*n* = 30)	*χ * ^2^/*P*
Nap habit			0.036/0.849
None	30 (58.82)	17 (56.67)	
Yes	21 (41.18)	13 (43.33)	
Sleeping time			1.980/0.577
<8 h	7 (13.73)	2 (6.67)	
8-9 h	32 (62.75)	19 (63.33)	
9-10 h	11 (21.57)	9 (30.00)	
>10 h	1 (1.96)	0 (0.0)	
Sleeping with the lights on at night			1.294/0.255
Yes	10 (19.61)	3 (10.00)	
No	41 (80.39)	27 (90.00)	
Outdoor light time			3.333/0.189
<1 h	14 (27.45)	14 (46.67)	
1-2 h	28 (54.90)	11 (36.67)	
>2 h	9 (17.65)	5 (16.67)	
Daily exercise time			**6.507/0.039**
<1 h	34 (66.67)	25 (83.33)	
1-2 h	15 (29.41)	2 (6.67)	
>2 h	2 (3.92)	3 (10.00)	
Daily use time of electronic products			**10.450/0.015**
0	4 (7.84)	2 (6.67)	
1-2 h	37 (72.55)	15 (50.00)	
2-3 h	10 (19.61)	8 (26.67)	
>3 h	0 (0.0)	5 (16.67)	
Romance TV dramas (movies)			**4.914/0.027**
Seen	9 (17.65)	12 (40.00)	
Never seen	42 (82.35)	18 (60.00)	
Adult skin care products (cosmetics)			—
Use	0 (0.0)	0 (0.0)	
Not used	51 (100.0)	30 (100.0)	

**Table 3:** Survey results of children's diet.

Project	Control group (*n* = 51)	Research group (*n* = 30)	*χ * ^2^/*P*
Frequency of drinking milk before half a year old			0.823/0.663
Breastfeeding	25 (49.02)	14 (46.67)	
Formula feeding	11 (21.57)	9 (30.00)	
Both	15 (29.41)	7 (23.33)	
Eating habits			1.060/0.589
Half and half meat and vegetable	26 (50.98)	13 (43.33)	
Meat-based	18 (35.29)	14 (46.67)	
Vegetarian-based	7 (13.73)	3 (10.00)	
Food intake			0.005/0.998
Too small	5 (9.80)	3 (10.00)	
Normal	31 (60.78)	18 (60.00)	
Larger	15 (29.41)	9 (30.00)	
Frequency of drinking milk			8.268/0.082
None	1 (1.96)	0 (0.0)	
1 time a week	10 (19.61)	8 (26.67)	
3-5 times a week	2 (3.92)	6 (20.00)	
1 time a day	27 (52.94)	9 (30.00)	
2 times a day or more	11 (21.57)	6 (20.00)	

**Table 4:** Survey results of children's family status.

Project	Control group (*n* = 51)	Research group (*n* = 30)	*χ * ^2^/*P*
Father's education level			2.930/0.403
Middle school and below	6 (11.76)	7 (23.33)	
High school	13 (25.49)	6 (20.00)	
College	25 (49.02)	11 (36.67)	
Master degree and above	7 (13.73)	6 (20.00)	
Father's profession			7.743/0.258
Service industry	6 (11.76)	1 (3.33)	
Sole proprietor	8 (15.69)	8 (26.67)	
Organs and institutions	7 (13.73)	5 (16.67)	
Corporate staff	7 (13.73)	7 (23.33)	
Professional technicians	16 (31.37)	5 (16.67)	
Migrant workers	3 (5.88)	0 (0.0)	
Other	4 (7.84)	4 (13.33)	
Mother's educational level			3.196/0.362
Middle school and below	5 (9.80)	5 (16.67)	
High school	16 (31.37)	6 (20.00)	
College	25 (49.02)	13 (43.33)	
Master degree and above	5 (9.80)	6 (20.00)	
Mother's profession			3.829/0.700
Service industry	6 (11.76)	1 (3.33)	
Sole proprietor	6 (11.76)	7 (23.33)	
Organs and institutions	7 (13.73)	4 (13.33)	
Corporate staff	8 (15.69)	5 (16.67)	
Professional technicians	10 (19.61)	5 (16.67)	
Migrant workers	1 (1.96)	0 (0.0)	
Other	13 (25.49)	8 (26.67)	
Monthly household income (yuan)			0.412/0.938
<0.5 million	5 (9.80)	3 (10.00)	
0.5–1.0 million	9 (17.68)	7 (23.33)	
1.0–2.0 million	18 (35.29)	10 (33.33)	
>2.0 million	19 (37.25)	10 (33.33)	
Children's family living environment			6.190/0.103
Separate room	33 (64.71)	12 (40.00)	
Share a room with parents	9 (17.65)	6 (20.00)	
Share a room with a brother (sister)	5 (9.80)	5 (16.67)	
Share a room with grandparents	4 (7.87)	7 (23.33)	
Parents marital status			**8.614/0.013**
Normal	49 (96.08)	22 (73.33)	
Divorced	2 (3.92)	7 (23.33)	
Remarry	0 (0.0)	1 (3.33)	
Family atmosphere			**6.188/0.045**
Very harmonious	21 (41.18)	6 (20.00)	
Normal	21 (41.18)	12 (40.00)	
Not good	9 (17.65)	12 (40.00)	
Father's accompaniment			**9.933/0.042**
None	0 (0.0)	2 (6.67)	
Rare	18 (35.29)	18 (60.00)	
Less than half	19 (37.25)	7 (23.33)	
More than half	8 (15.69)	2 (6.67)	
Most	6 (11.76)	1 (3.33)	
Mother's accompaniment			**11.300/0.010**
None	0 (0.0)	0 (0.0)	
Rare	3 (5.88)	6 (20.00)	
Less than half	6 (11.76)	6 (20.00)	
More than half	6 (11.76)	8 (26.67)	
Most	36 (70.59)	10 (33.33)	

**Table 5:** Survey results of children's physiological status.

Project	Control group (*n* = 51)	Research group (*n* = 30)	*χ * ^2^/*P*
Difficulty walking more than 200 meters			5.664/0.129
There has never been	45 (88.24)	21 (70.00)	
Almost none	5 (9.80)	5 (16.67)	
Sometimes	1 (1.96)	3 (10.00)	
Frequently	0 (0.0)	0 (0.0)	
Always	0 (0.0)	1 (3.33)	
Difficulty running			3.555/0.314
There has never been	36 (70.59)	16 (53.33)	
Almost none	7 (13.73)	9 (30.00)	
Sometimes	7 (13.73)	4 (13.33)	
Frequently	0 (0.0)	0 (0.0)	
Always	1 (1.96)	1 (3.33)	
Difficulty participating in sports or exercise			3.590/0.464
There has never been	33 (64.71)	16 (53.33)	
Almost none	11 (21.57)	6 (20.00)	
Sometimes	5 (9.80)	6 (20.00)	
Frequently	1 (1.96)	2 (6.67)	
Always	1 (1.96)	0 (0.0)	
Difficulty lifting heavy objects			7.695/0.103
There has never been	35 (68.63)	12 (40.00)	
Almost none	9 (17.65)	11 (36.67)	
Sometimes	3 (5.88)	5 (16.67)	
Frequently	2 (3.92)	1 (3.33)	
Always	2 (3.92)	1 (3.33)	
Difficulty taking a bath			6.440/0.092
There has never been	41 (80.39)	21 (70.00)	
Almost none	4 (7.84)	8 (26.67)	
Sometimes	5 (9.80)	1 (3.33)	
Frequently	0 (0.0)	0 (0.0)	
Always	1 (1.96)	0 (0.0)	
Difficulty doing housework			5.632/0.131
There has never been	35 (68.63)	17 (56.67)	
Almost none	4 (7.84)	8 (26.67)	
Sometimes	8 (15.69)	4 (13.33)	
Frequently	4 (7.84)	1 (3.33)	
Always	0 (0.0)	0 (0.0)	
Injuries or pain			6.648/0.156
There has never been	27 (52.94)	13 (43.33)	
Almost none	15 (29.41)	6 (20.00)	
Sometimes	7 (13.73)	11 (36.67)	
Frequently	1 (1.96)	0 (0.0)	
Always	1 (1.96)	0 (0.0)	
Poor physical strength			7.652/0.054
There has never been	32 (62.75)	13 (43.33)	
Almost none	14 (27.45)	8 (26.67)	
Sometimes	4 (7.84)	9 (30.00)	
Frequently	1 (1.96)	0 (0.0)	
Always	0 (0.0)	0 (0.0)	

**Table 6:** Survey results of parents' psychological states.

Project	Control group (*n* = 51)	Research group (*n* = 30)	*χ * ^2^/*P*
Feeling exhausted			**8.952/0.030**
There has never been	16 (31.37)	7 (23.33)	
Almost none	17 (33.33)	3 (10.00)	
Sometimes	15 (29.41)	18 (60.00)	
Frequently	3 (5.88)	2 (6.67)	
Always	0 (0.0)	0 (0.0)	
Feeling of headache			1.446/0.695
There has never been	19 (37.25)	11 (36.67)	
Almost none	14 (27.45)	9 (30.00)	
Sometimes	17 (33.33)	8 (26.67)	
Frequently	1 (1.96)	2 (6.67)	
Always	0 (0.0)	0 (0.0)	
Feeling of weakness			5.731/0.220
There has never been	24 (47.06)	10 (33.33)	
Almost none	15 (29.41)	12 (40.00)	
Sometimes	11 (21.57)	5 (16.67)	
Frequently	0 (0.0)	2 (6.67)	
Always	1 (1.96)	0 (0.0)	
Feeling of nausea			0.003/0.999
There has never been	27 (52.94)	16 (53.33)	
Almost none	19 (37.25)	11 (36.67)	
Sometimes	5 (9.80)	3 (10.00)	
Frequently	0 (0.0)	0 (0.0)	
Always	0 (0.0)	0 (0.0)	
Feeling of anxiety			**16.020/0.003**
There has never been	22 (43.14)	3 (10.00)	
Almost none	7 (13.73)	2 (6.67)	
Sometimes	18 (35.29)	19 (63.33)	
Frequently	4 (7.84)	3 (10.00)	
Always	0 (0.0)	3 (10.00)	
Feeling of sadness			**14.230/0.003**
There has never been	21 (41.18)	4 (13.33)	
Almost none	13 (25.49)	5 (16.67)	
Sometimes	16 (31.37)	15 (50.00)	
Frequently	1 (1.96)	6 (20.00)	
Always	0 (0.0)	0 (0.0)	
Feeling of anger			**11.700/0.009**
There has never been	20 (39.22)	4 (13.33)	
Almost none	12 (23.53)	9 (30.00)	
Sometimes	18 (35.29)	11 (36.67)	
Frequently	1 (1.96)	6 (20.00)	
Always	0 (0.0)	0 (0.0)	
Feeling of depression			**8.238/0.041**
There has never been	23 (45.10)	7 (23.33)	
Almost none	12 (23.53)	9 (30.00)	
Sometimes	15 (29.41)	9 (30.00)	
Frequently	1 (1.96)	5 (16.67)	
Always	0 (0.0)	0 (0.0)	
Feeling of helplessness			**8.815/0.032**
There has never been	24 (47.06)	8 (26.67)	
Almost none	18 (35.29)	9 (30.00)	
Sometimes	8 (15.69)	8 (26.67)	
Frequently	1 (1.96)	5 (16.67)	
Always	0 (0.0)	0 (0.0)	

## Data Availability

The dataset used and/or analyzed during the current study are available from the corresponding author.
